The article "Association of Cytokine Gene Polymorphisms with Prostate Cancer Risk from a Study in Central China" was published in 2022. Journal: Contrast Media Mol Imaging.

# Association of Cytokine Gene Polymorphisms with Prostate Cancer Risk from a Study in Central China

**DOI:** 10.1155/2022/1259009

**Published:** 2022-08-13

**Authors:** Shun Xu, Yongtao Hu, Ligang Zhang, Shaoyu Yue, Li Zhang, Chaozhao Liang

**Affiliations:** ^1^Department of Urology, The First Affiliated Hospital of Anhui Medical University, Hefei, China; ^2^Institute of Urology, Anhui Medical University, Hefei, China; ^3^Anhui Province Key Laboratory of Genitourinary Diseases, Anhui Medical University, Hefei, China

## Abstract

Our study intended to investigate five cytokine gene single nucleotide polymorphisms (SNPs) and their associations with prostate cancer risk. Genotypes of five cytokine gene SNPs were detected by MassARRAY for blood samples from a group of patients with prostate cancer (*n* = 90) and a control group (*n* = 140) in central China. The differences in tumor clinical stages, Gleason scores, and PSA values in patients with prostate cancer were also investigated. The frequencies of the five cytokine gene SNPs (L-1*β* rs16944, IL-4 rs2070874, IL-4rs2227284, IL-16 rs7175701, and IL-16 rs11556218) genotypes were not found to be significantly mutated in prostate cancer patients compared with the control group. In addition, for five cytokine gene SNPs genotypic comparisons, patients with different Gleason scores, clinical stages, and PSA values were grouped into two subgroups. There was also no statistically significant association in all these subgroups. Our study suggests that cytokine gene polymorphisms may not be a risk factor for prostate cancer in a central Chinese population. Nevertheless, more large-scale studies on the Chinese population are necessary to examine our conclusions. The discovery of cytokine gene polymorphisms related to prostate cancer could update our understanding of the etiology and improve our knowledge of the early detection, diagnosis, and treatment of prostate cancer.

## 1. Introduction

Prostate cancer (PCa) is the most common urinary neoplasm in men, which is estimated to account for about 21% of all cases of newly diagnosed cancers and account for 33,330 cases of deaths in males in America [1]. Although the incidence of prostate cancer in Asian populations is low, the incidence continues to rise. Like other cancers, the pathogenesis and tumorigenesis of prostate cancer are still not clear to the public [2]. Up till now, many factors, including ethnicity, age, or family history, have been identified to affect the incidence of prostate cancer [3]. In addition, lifestyle behaviors [4–6] and even genetic factors [7–10] were also regarded as risk factors for prostate cancer. Furthermore, studies have demonstrated that the morbidity of PCa is gene-related at a level of approximately 57% [11], and of those, inflammation-related genes are extensively studied. The diagnosis of prostate cancer is based on a microscopic evaluation of prostate tissue obtained through a needle biopsy. Conventionally, a systematic prostate biopsy is performed using transrectal ultrasound to obtain 10 to 12 gridded tissue samples. Pathologists examine these samples and assign a primary Gleason grade for the predominant histological pattern and a secondary grade for the highest pattern, both on a scale of 1 to 5, based on the microstructure and appearance of the cells. Clinicians have traditionally classified diagnoses as low-risk, intermediate-risk, and high-risk based on the sum of the Gleason pattern, prostate-specific antigen (PSA) level, and clinical stage [12]. Therapeutic methods for prostate cancer, in which surgery and radiation therapy remain treatments for localized disease, but have side effects such as urinary symptoms and sexual dysfunction that negatively impact the quality of life. For metastatic disease, chemotherapy as initial therapy now appears to prolong survival compared with androgen deprivation therapy alone. New vaccines, hormone therapy, and bone-targeting agents have been shown to be effective in men with metastatic prostate cancer resistant to conventional hormone therapy [12, 13].

Infections and inflammatory responses have been reported to be associated with approximately 15% of cancer deaths globally. Chronic inflammation was considered to have an important role in the pathogenetic process of cancers [14, 15] and is now relevant to the early steps of oncogenesis and cancer progression [16, 17]. Inflammation of the prostate was reported to participate in the occurrence and development of prostate cancer [18, 19]. The features of cancer-related inflammation include the infiltration of white blood cells and the production of inflammatory mediators accompanying chronic inflammation, which is often observed in the process of tissue reconstruction and repair [16]. One of the most important components of the inflammatory mediators is the production of cytokines associated with the host immune response. Therefore, genetic variability in altering gene expressions within key cytokines may be related to prostate cancer risk. Cytokine gene single nucleotide polymorphisms (SNPs) of interleukin (IL)-1*β*, IL-4, and IL-16 genes have been reported to be associated with the risk of cancers, including renal cell carcinoma, gastric carcinoma, and lung cancer [20–22]. For PCa, some studies reported that interleukin gene polymorphisms may contribute to the occurrence of prostate cancer [23–25]. For example, Luo et al. reported that IL-4 SNPs in PCa were related to cancer risk or mortality [26]. Shailendra Dwivedi et al. concluded that genetic variants of IL-18 and IL-10 promoters influence the circulating levels of these interleukins. Variations at −137 and −607 loci of IL-18 are associated with susceptibility to PCa [27]. Prostate tumor cells produce large amounts of IL-6 and its receptor, IL-6R (gp80), and IL-6 functions as a paracrine growth factor for the human LNCaP androgen-sensitive prostate cancer cells and an autocrine growth factor for the human DU145 and PC3 androgen-insensitive prostate cancer cells [28–32].

However, some other studies reported that there is no association observed between interleukin gene polymorphisms and prostate cancer [33, 34]. Thus, the association between candidate cytokine gene SNPs and prostate cancer remains to be an unsettled issue.

In this study, we intend to investigate the association between the cytokine gene SNPs genotypes and allele distributions and prostate cancer risk. IL-1*β* and IL-16 gene SNPs were designed for their role in promoting inflammation, and IL-4 gene SNPs were designed for their role in suppressing inflammation. These polymorphisms have been studied before with conflicting results. However, few studies have been conducted on Asian populations, especially in China. Therefore, to figure out the association between the cytokine gene SNPs and prostate cancer risk, we performed this hospital-based case-control study to validate the risk of five cytokine gene SNPs on prostate cancer.

## 2. Materials and Methods

### 2.1. Study Subjects

This study was performed according to the Declaration of Helsinki and approved by the Ethics Committee of the first affiliated hospital of Anhui Medical University, Hefei, Anhui, China. All patients or participants signed written informed consent to allow analysis of data for research use. In this study, we adopted a value of Cohen's *d* of 0.7, a statistical power level of 0.8, and a *p* value as 0.05. After calculation, the minimum total sample size was 52 in the evaluation and a minimum sample size of 26 for each group. Totally, between September 2014 and July 2016, ninety patients newly diagnosed with prostate cancer who underwent prostate biopsy were included in this study. Patients with prostate cancer were subdivided into two groups according to Gleason score (low grade ≤ 7 and high grade > 7), clinical stages (based on the international tumor node-metastasis system for PCa, localized and advanced), and PSA values (PSA ≤ 20 ng/ml and PSA > 20 ng/ml). Correspondingly, 140 volunteers were recruited into a healthy control group from individuals who came to the hospital for a routine health examination. All of the healthy people were included according to the following criteria: normal physical examination indicators; no genetic family history; no diagnosis of acute infectious diseases; no drinking or smoking habits; no history of drug abuse; and no impairment of the liver, heart, or kidney. All of the PCa patients were included according to the following criteria: no history of cancer or prostate surgery; no diagnosis of acute infectious diseases; no therapeutic medication for PCa; and no impairment of the liver, heart, or kidney. Venous blood samples were collected from all the participants after fasting for at least 12 hours. We also gathered related clinical and pathological data, including body mass index (BMI), systolic blood pressure (SBP), and serum PSA values from the medical record.

### 2.2. Selection of SNPs for Evaluation and Genotyping

The total DNA of all patients and controls was extracted from venous blood samples by using commercial DNA extraction kits (Qiagen, # 51106). In the study, we selected five cytokine gene SNPs through the SNP Consortium database (https://snp.cshl.org/) and the DbSNP database (https://www.hapmap.org/index.html.en) for analysis, and each SNP had a minor allele frequency (MAF) of >5% in the Chinese Han population. The five cytokine gene SNPs included *L-*1*β* rs16944, IL-4 rs2070874, IL-4rs2227284, IL-16 rs7175701, and IL-16 rs11556218. For each DNA sample, five cytokine gene polymorphisms were detected by MassARRAY (Sequenom, San Diego, USA). Details of the experiment process are referred to in Qin et al.'s [35] study. The data were analyzed by TYPER 4.0 software (Sequenom).

### 2.3. Statistical Analysis

The Hardy-Weinberg equilibrium (HWE) of cases and controls were calculated by chi-square analysis. The cancer risk, which was assessed by ORs with 95% CI, was calculated by using logistic regression models; otherwise, calculation results were adjusted for age and BMI. *P* < 0.05 was identified to be statistically significant. The differences in tumor clinical stages, Gleason scores, and PSA values in patients with prostate cancer were also investigated by using the statistical methods mentioned above. The software used for statistical analyses in the study was IBM SPSS Statistics 20.0 (IBM Corp., Armonk, NY, USA).

## 3. Results

### 3.1. Characteristics of the Study Subjects

Table 1 showed the detailed demographic characteristics of study subjects. The mean age of PCa patients was 73.00 years old, ranging from 48 to 87 years. The mean age of the controls was 67.66 years old, ranging from 60 to 95 years. Between the two groups, we found a significant difference in age (*P* < 0.001). According to the World Health Organization recommendations for Asian populations, the normal BMI range is 18.5–22.9 kg/m2. There were no significant differences in BMI and systolic blood pressure between the PCa group and the control group. PCa patients were divided into two groups by PSA, Gleason score, and tumor clinical stage, respectively.

### 3.2. Association of Five Cytokine Gene SNPs with Prostate Cancer Risk

All five cytokine gene SNPs were in HWE among the PCa group and the control group (*P* > 0.05). The genotypic distributions and allele frequencies of cytokine gene SNPs between the two groups are described in Table 2. Stratification analyses of genotypes on risk of PCa were performed by age, BMI, and SBP groups (Table 3). Then, we performed a comparative analysis of genotypes in PCa patients. These patients were subdivided into two groups according to different Gleason scores (Gleason score ≤ 7, low-grade group; Gleason score > 7, high-grade group), TNM staging (localized group and advanced group), and PSA levels (PSA ≤ 20 group; PSA > 20 group), respectively (Table 4). The details of the results of five cytokine gene SNPs are listed below:

### 3.3. IL-1*β* rs16944

The IL-1*β* rs16944 genotypic distributions of the control group complied with HWE (*P*=0.120). There was no difference between the PCa patients and the control group in the frequencies of rs16944 genotypes, including GG, GA, and AA (Table 2). Compared with GG, the variant GA and AA genotypes were not associated with the risk of prostate cancer after an adjustment of age and BMI (GA vs. GG: adjusted OR = 0.689, 95% CI (0.335, 1.418), *P*=0.097; AA vs. GG: adjusted OR = 0.734, 95% CI (0.316, 1.701), *P*=0.694; GA + AA vs. GG: adjusted OR = 0.705, 95% CI (0.361, 1.379), *P*=0.188). When analyzing frequencies of haplotypes, compared to *G* allele, the variant A allele was also not associated with PCa risk (*P*=0.771). In addition, stratification analyses showed that when grouped by age, compared to GG genotypes, the variant AG (*P*=0.019) and AG + AA (*P*=0.041) genotypes showed a protective role for prostate cancer in the age > 70 group. There was also no significant difference in the stratified analysis results of different BMI groups and SBP groups (Table 3).

### 3.4. IL-4 rs2070874

The *IL-4* rs2070874 genotypic distributions of the control group complied with HWE (*P*=0.751*P*=0.751). The distributions of rs2070874 genotypes were similar between the PCa group and the control group (Table 2). Compared with TT, the variant TC and CC genotype were not associated with the risk of prostate cancer after adjusting for age and BMI (TC vs. TT: adjusted OR = 1.159, 95% CI (0.637, 2.109), *P*=0.528; CC vs. TT: adjusted OR = 0.314, 95% CI (0.034, 2.896), *P*=0.285; TC + CC vs. TT: adjusted OR = 1.072, 95% CI (0.597, 1.924), *P*=0.707). When analyzing frequencies of haplotypes, compared to *T* allele, the variant C allele was also not a risk for prostate cancer (*P*=1.000). In addition, stratification analysis showed that there was no significant difference in age, BMI, and SBP groups (Table 3).

### 3.5. IL-4 rs2227284

The *IL-*4 rs2227284 genotypic distributions of the control group complied with HWE (*P*=0.176). The distributions of rs2227284 genotypes were similar between the PCa group and the control group (Table 2). Compared with TT genotypes, the variant TG and GG genotypes do not affect the risk of prostate cancer after an adjustment of age and BMI(TG vs. TT: adjusted OR = 0.669, 95% CI: (0.343, 1.304), *P*=0.347; GG vs. TT: adjusted OR = 2.718, 95% CI: (0.155,47.524), *P*=0.793; TG + GG vs. TT: adjusted OR = 0.703, 95% CI: (0.365,1.355), *P*=0.380). As for the alleles, compared to *T* allele, the variant *G* allele does not influence the risk of prostate cancer (*p*=0.461). In addition, stratified analyses showed that when grouped by age, compared with TT, the variant TG (*P*=0.031) genotypes could decrease the risk of prostate cancer in age ≤ 70 group. There was also no significant difference in the stratified analysis results of different BMI groups and SBP groups (Table 3).

### 3.6. IL-16 rs7175701

The *IL-1*6 rs7175701 genotypic distributions of the control group complied with HWE (*P*=0.694). The distributions of rs7175701 genotypes were similar between the PCa group and the control group (Table 2). Compared with TT, the variant TC genotype does not affect the risk of prostate cancer after an adjustment of age and BMI (TC vs. TT: adjusted OR = 0.224, 95% CI (0.044, 1.143), *P*=0.145). As for the alleles, compared to *T* allele, the variant C allele does not influence the risk of prostate cancer (*p*=0.150). Besides, stratification analysis showed that there was no significant difference in age, BMI, and SBP groups (Table 3).

### 3.7. IL-16 rs11556218

The IL-16 rs11556218 genotypic distributions of the control group complied with HWE (*P*=0.604). The distributions of rs11556218 genotypes were similar between the PCa group and the control group (Table 2). Compared to TT, the variant TG and GG genotypes do not affect the risk of prostate cancer after an adjustment of age and BMI (TG vs. TT: adjusted OR = 0.507), 95% CI: (0.264, 0.976), *P*=0.053; GG vs. TT: adjusted OR = 0.598, 95% CI: (0.138, 2.588), *P*=0.979; TG + GG vs. TT: adjusted OR = 0.525, 95% CI: (0.281, 0.978), *P*=0.079. As for the alleles, compared to *T* allele, the variant *G* allele showed no association with the risk of prostate cancer (*P*=0.166). In addition, stratified analyses showed that when grouped by age, compared with TT, the variant TG (*P*=0.029) genotypes could decrease the risk of prostate cancer in age > 70 group. No significant differences were also found by stratification analysis when performed by BMI and SBP groups (Table 3).

Distributions of the five cytokine gene SNPs genotypes in patients with prostate cancer were also analyzed. PCa patients with different Gleason scores, clinical stages, and PSA values were subdivided into two groups. As a result, there were no significant differences in the five cytokine gene SNPs genotypic frequencies by Gleason scores, clinical stages, and PSA levels (Table 4).

## 4. Discussion

Like many other tumors, the cause of prostate cancer is unknown. Numerous factors have been reported to increase the incidence of cancer. In recent years, many studies have reported that there may be a link between gene polymorphisms and PCa risks. From then on, subsequent studies have demonstrated SNPs could affect the occurrence of PCa [36, 37]. Interestingly, inflammation has been suggested as a potential trigger for the development of prostate cancer [38]. Epidemiological studies have demonstrated this viewpoint, and the use of anti-inflammatory agents could decrease the risk of prostate cancer [39]. Thus, we hold the opinion that the variants in relevant genes encoding certain proinflammatory or anti-inflammatory cytokines may affect prostate cancer risk since cytokine gene SNPs could lead to aberrant expression of cytokines [40, 41].

IL-1*β* is a 17-kDa cytokine member of the interleukin-1 family, which is involved in inflammation and immunity. The IL-1*β* gene is located on chromosome 2q14, and its expression has been reported to be related to different diseases [42, 43]. *IL-*1*β* gene polymorphisms are associated with increased secretion of cytokine IL-1*β* when compared to the wild-type gene [40]. In recent years, it has been reported that *IL*-1*β* gene polymorphisms may be related to various cancer types, including gastric carcinoma [21], hepatic carcinoma [44], and lung cancer [45].

IL-4 is a member of the *α*-helical cytokine family, which is secreted by activated CD4+ T cells, basophils, and mast cells. IL-4 is an important component of our immune system and is involved in functions such as inhibition of the production of proinflammatory cytokines by monocytes and immunoglobulin class switching in activated B lymphocytes. Thus, IL-4 plays a vital role in the inhibition of inflammation and the surveillance and elimination of transformed cells. Many epidemiologic studies have reported the association of IL-4 gene SNPs with cancer risks, such as breast cancer [46], gastric cancer [47], and lung cancer [22].

IL-16 is a proinflammatory cytokine that has a wide array of functions in multiple immunopathobiological processes [48]. IL-16 stimulates the production of a variety of proinflammatory cytokines by monocytes with related biological sequelae [49]. Evidence of increased IL-16 levels in serum or plasma has also been recognized in multiple malignant tumors in both preclinical and clinical trials [50–52]. Studies have reported a relationship between IL-16 gene polymorphisms and cancers, including gastric cancer [53], renal cell cancer [20], and colorectal cancer [54].

For PCa, previous studies reported that IL-1*β*, IL-4, and IL-16 gene polymorphisms could affect the incidence of prostate cancer [24, 25, 55]. The five cytokine gene SNPs we selected in this study were hardly investigated, especially in China. In the present study conducted in central China, we found that all these five cytokine-related loci, including *I*L-1*β* rs16944, IL-4 rs2070874, IL-4 rs2227284, IL-16 rs7175701, and IL-16 rs11556218 were all not significantly associated with the occurrence of prostate cancer. The results of the present study were inconsistent with previous studies reported on the Turkish and African American populations. Faruk Yencilek et al. showed that individuals with the IL1B-31 (rs1143627) and IL1B-511 (rs16944) AG genotypes have a reduced risk of prostate cancer. Of all possible combinations analyzed, the combination of IL1B-31 (rs1143627) *G* and IL1B-511 (rs16944) *G* prevented the development of prostate cancer. To the best of our knowledge, the data obtained in this study are the first to highlight the association of IL1B gene variants with prostate cancer in the Turkish population [55]. Meanwhile, in prostatectomy tumor specimens of prostate cancer patients, the expression of IL-16 is positively correlated with Gleason score and pathological stage, and IL-16 is also highly expressed in other types of tumor cells. The level of IL-16 in serum is also elevated in patients with other types of cancer, especially in patients with advanced cancer. Ken Batai et al. provide evidence that IL-16 polymorphisms show great significance in Pca susceptibility in African Americans. To our knowledge, this is the first study that demonstrated the association of these variants with cancer in African-descent populations [25]. However, our study suggests that the effect of the five cytokine gene SNPs on PCa may have a racial difference in different populations, though further investigations will be needed.

Additionally, we conducted the analysis of genotypes comparison in PCa patients. These patients were subdivided into two groups according to different Gleason scores (Gleason score ≤ 7, low-grade group; Gleason score > 7, high-grade group), TNM staging (localized group and advanced group), and PSA levels (PSA ≤ 20 group; PSA > 20 group), respectively. As a result, there was no significant association observed between the cytokine gene polymorphisms and all these subgroups of prostate cancer. Our study suggested that the five cytokine gene SNPs may not be related to cancer progression in prostate cancer.

However, there were some limitations to our study. Firstly, although our participants were recruited from a relatively homogenous Chinese population in Anhui province, a central area of China, we could not thoroughly eliminate the influence of potential genetic background. Secondly, for the case-control study, the sample size may be a limitation. Thirdly, the lack of an independent set of samples to examine our conclusions is another limitation. Thus, we plan to carry out further optimization studies and pay attention to the following issues: first of all, when we screen patients, we investigate their genetic backgrounds to ensure that they are as similar as possible. Second, the age difference between the control group and the case group should be minimized. Finally, select a few provinces in central China, not just Anhui, so that it is representative and the sample size is large enough.

Thus, further large-sample studies should be conducted on Chinese populations to evaluate our results. In addition, the age difference between the cases and control group may affect the results of our study.

Bioinformatics is an emerging discipline that emerged with the launch of the Human Genome Project (HGP), which integrates mathematics, computer science, and biology to elucidate the biological significance of various types of data. Currently, bioinformatics plays a pivotal role in the development of medicine. First, based on different omics datasets such as transcriptome, proteome, and epigenome, using clustering, consensus, and other ideas to achieve disease classification is of great significance for understanding the disease mechanism. [56–59] In addition, bioinformatics can be used to predict and analyze gene variants, expression, as well as gene and protein structure and function, which are crucial for disease diagnosis and treatment. Therefore, in the future, we should combine immunological therapy with bioinformatics to deeply research the pathology of diseases.

## 5. Conclusion

In summary, the present study suggests that cytokine gene polymorphisms, including IL-1*β* rs16944, IL-4 rs2070874, IL-4 rs2227284, IL-16 rs7175701, and IL-16 rs11556218 may not be risk factors for prostate cancer in a population in central China. Nevertheless, more large-scale studies on the Chinese population are necessary to examine our conclusions. The discovery of prostate cancer-related cytokine gene polymorphisms could update our understanding of the etiology and improve our knowledge of the early detection, diagnosis, and treatment of prostate cancer.

## Figures and Tables

**Table 1:** Characteristics of prostate cancer cases and controls in central China.

Characteristic	Control	PCa case	*P* value^a^	Or (95% CI)
Sample size	*n* = 140	*n* = 90		
Age (years ± SD)	67.66 ± 6.69	73.00 ± 7.64	<0.001	
Age years			<0.001	3.715 (2.128–6.487)
≤70	97	34		
>70	43	56		
BMI			0.098	1.661 (0.910–3.030)
≤23	47	21		
>23	93	69		
SBP			0.787	1.076 (0.633–1.827)
<140	71	44		
≥140	69	46		
PSA ng/mL				
≤20	—	51	—	—
>20	—	39	—	—
Gleason score				
>7	—	36	—	—
≤7	—	54	—	—
Tumor clinical stage				
Localized	—	68	—	—
Advanced	—	22	—	—

Notes: ^a^Two-sided *x*^2^ test for the distributions between the cases and controls. PCa, prostate cancer; BMI, body mass index; SBP, systolic blood pressure.

**Table 2:** Association of cytokine gene SNPs with prostate cancer risk in central China.

Gene	Position	dbSNP ID			Prostate cancer cases (*N* = 90)	Controls (*N* = 140)	*P* Value	Or (95% CI)	Adjusted OR (95% CI)^b^	HWE^c^	HWE^d^
IL-1*β*	2:112837290	rs16944	Genotypes	GG	24	27		1 (reference)		0.120	0.294
				GA	40	79	0.097	0.570 (0.292, 1.112)	0.689 (0.335, 1.418)		
				AA	26	34	0.694	0.860 (0.406, 1.822)	0.734 (0.316, 1.701)		
				GA + AA	66	113	0.188	0.657 (0.351, 1.231)	0.705 (0.361, 1.379)		
			Alleles	G	88	133		1 (reference)			
				A	92	147	0.771	0.946 (0.650, 1.376)			

IL-4	5:132674018	rs2070874	Genotypes	TT	55	89		1 (reference)		0.751	0.087
				TC	34	46	0.528	1.196 (0.686, 2.086)	1.159 (0.637, 2.109)		
				CC	1	5	0.285	0.324 (0.037, 2.844)	0.314 (0.034, 2.896)		
				CT + CC	35	51	0.707	1.111 (0.643, 1.917)	1.072 (0.597, 1.924)		
			Alleles	T	144	224		1 (reference)			
				C	36	56	1.000	1.000 (0.626, 1.597)			

IL-4	5:132677033	rs2227284	Genotypes	TT	69	100		1(reference)		0.176	0.735
				TG	20	39	0.347	0.743 (0.400, 1.382)	0.669 (0.343, 1.304)		
				GG	1	1	0.793	1.449 (0.089, 23.566)	2.718 (0.155, 47.524)		
				TG + GG	21	40	0.380	0.761 (0.413, 1.401)	0.703 (0.365, 1.355)		
			Alleles	T	158	239		1 (reference)			
				G	22	41	0.461	0.812 (0.466, 1.415)			

IL-16	15:81266282	rs7175701	Genotypes	TT	88	131		1 (reference)		0.694	0.915
				TC	2	9	0.145	0.331 (0.070, 1.568)	0.224 (0.044, 1.143)		
				CC	0	0	—	—	—		
				TC + CC	2	9	0.145	0.331 (0.070, 1.568)	0.224 (0.044, 1.143)		
			Alleles	T	178	271		1 (reference)			
				C	2	9	0.150	0.388 (0.072, 1.584)			

IL-16	15:81305928	rs11556218	Genotypes	TT	66	87		1 (reference)			
				TG	20	48	0.053	0.549 (0.298, 1.013)	0.507 (0.264, 0.976)	0.604	0.144
				GG	4	5	0.979	1.018 (0.263, 3.942)	0.598 (0.138, 2.588)		
				TG + GG	24	53	0.079	0.597 (0.335, 1.065)	0.525 (0.281, 0.978)		
			Alleles	T	152	222		1 (reference)			
				G	28	58	0.166	0.705 (0.429, 1.158)			

Notes: ^a^Two-sided *x*^2^ test for the distributions between the cases and controls; ^b^adjusting for age and body mass index (BMI); ^c^Hardy Weinberg Equilibrium in controls; ^d^Hardy Weinberg Equilibrium in cases.

**Table 3:** Stratification analysis of genotypes and risk of PCa conducted by age, BMI, and SBP.

	AA (case/Control)	AB (case/Control)	BB (case/Control)	AB + BB (case/Control)	*P*1	OR1 (95% CI)	*P*2	OR2 (95% CI)	*P*3	OR3 (95% CI)
rs16944	GG	AG	AA	AG + AA						
Age	24/27	40/79								
≤70	6/21	20/55	7/21	27/176	0.650	1.273 (0.499, 3.607)	0.808	1.167 (0.335, 4.060)	0.671	1.243 (0.454–3.407)
>70	18/6	20/24	19/13	39/137	**0.019**	0.287 (0.093, 0.833)	0.222	0.487 (0.152, 1.558)	**0.041**	0.351 (0.126–0.982)
BMI										
≤23	3/8	10/30	8/9	18/39	1.000	0.889 (0.197, 4.014)	0.515	2.370(0.463, 12.138)	1.000	1.231 (0.292–5.193)
>23	21/19	30/49	18/25	48/74	0.130	0.559 (0.257, 1.195)	0.332	0.651 (0.274, 1.551)	0.144	0.587 (0.286, 1.205)
SBP										
<140	12/17	20/40	13/14	33/54	0.458	0.708 (0.284, 1.766)	0.611	1.315 (0.457, 3.783)	0.741	0.866 (0.368, 2.039)
≥140	12/10	20/39	13/30	33/59	0.091	0.427 (0.158, 1.159)	0.269	0.542 (0.182, 1.614)	0.107	0.466 (0.182, 1.195)

rs2070874	TT	TC	CC	TC + CC						
Age	55/89	34/46	1/5	35/51						
≤70	23/58	10/36	1/3	11/39	0.411	0.700 (0.299, 1.640)	1.000	0.841 (0.083, 8.503)	0.417	0.711 (0.312, 1.623)
>70	32/31	24/10	0/2	24/12	0.060	2.325 (0.957, 5.649)	0.492	2.032 (.581, 2.612)	0.125	1.938 (0.827, 4.537)
BMI										
≤23	16/32	4/14	0/1	20/25	0.233	1.597 (0.738, 3.456)	1.000	1.522 (1.285, 1.802)	0.274	1.533(0.712, 3.304)
>23	39/57	30/32	1/4	15/26	0.764	0.833 (0.391, 1.992)	0.621	0.347 (0.037, 3.256)	0.578	0.800 (0.365, 1.755)
SBP										
<140	24/46	20/24	0/1	20/25	0.233	1.597 (0.738, 3.456)	1.000	1.522 (1.285, 1.802)	0.274	1.533 (0.712, 3.304)
≥140	31/43	14/22	1/4	15/26	0.764	0.883 (0.391, 1.992)	0.621	0.347 (0.037, 3.256)	0.578	0.800(0.365, 1.755)

rs2227284	TT	TG	GG	TG + GG						
Age	69/100	20/39	1/1							
≤70	29/66	4/30	1/1	5/31	**0.031**	0.303 (0.098, 0.940)	0.525	2.276 (0.138, 37.651)	0.052	0.367 (0.130, 1.039)
>70	40/34	16/9	0/0	16/9	0.386	1.511 (0.593, 3.853)	—	—	0.386	1.511 (0.593, 3.853)
BMI										
≤23	17/37	3/9	0/1	3/10	0.925	0.725 (0.174, 3.023)	1.000	1.459 (1.218, 1.749)	0.797	0.653 (0.159, 2.680)
>23	52/63	17/30	1/0	18/30	0.291	0.687(0.341, 1.381)	0.457	2.212(1.809, 2.704)	0.364	0.727(0.365, 1.450)
SBP										
<140	35/54	9/17	0/0	9/17	0.664	0.817 (0.328, 2.035)	—	—	0.664	0.817 (0.328, 2.035)
≥140	34/46	11/22	1/1	12/23	0.365	0.676 (0.290, 1.581)	1.000	1.353 (0.082, 22.406)	0.408	0.706 (0.309, 1.614)

rs7175701	TT	TC	CC	TC + CC						
Age	88/131	2/9								
≤70	31/193	1/4	0/0	¼	1.000	0.750 (0.081, 6.966)	—	—	—	—
>70	57/138	1/5	0/0	1/5	0.098	0.133 (0.015, 1.187)	—	—	—	—
BMI										
≤23	20/45	0/2	0/0	0/2	1.000	1.444 (1.228, 1.699)	—	—	—	—
>23	68/86	2/7	0/0	2/7	0.334	0.361 (0.073, 1.796)	—	—	—	—
SBP										
<140	43/67	2/4	0/0	2/4	1.000	0.779 (0.137, 4.439)	—	—	—	—
≥140	45/64	0/5	0/0	0/5	0.168	1.703 (1.155, 1.993)	—	—	—	—

rs11556218	TT	TG	GG	TG + GG						
Age	66/87	20/48	4/5							
≤70	24/63	9/31	0/3	9/34	0.544	0.762 (0.317, 1.835)	0.562	1.381 (1.213–1.572)	0.412	0.695 (0.270–1.662)
>70	42/24	11/17	4/2	15/19	**0.029**	0.370 (0.149–0.918)	1.000	1.143 (0.195–6.709)	0.062	0.451 (0.194–1.048)
BMI										
≤23	15/32	4/15	1/0	5/15	0.378	0.569 (0.161–2.010)	0.269	6.290 (0.242–163.426)	0.571	0.711 (0.218–2.322)
>23	5/55	16/33	3/5	19/38	0.071	0.523 (0.258–1.062)	0.822	0.647 (0.147–2.846)	0.069	0.539 (0.276, 1.053)
SBP										
<140	34/45	8/23	3/3	11/26	0.094	0.460 (0.184–1.155)	1.000	1.324 (0.251–6.969)	0.170	0.560 (0.243–1.289)
≥140	32/42	12/25	1/2	13/27	0.272	0.630 (0.275–1.442)	1.000	0.656 (0.057–7.560)	0.263	0.632 (0.282–1.415)

Notes: *P*1, OR1: comparison between AB vs. AA; *P*2, OR2: comparison between BB vs. AA; *P*3, OR3: comparison between AB + BB vs. AA. PCa, prostate cancer; BMI, body mass index; SBP, systolic blood pressure.

**Table 4:** Cytokine gene polymorphisms and clinic pathological characteristics with the PCa patients in central China.

	AA	AB + BB	*P* value^a^	Or (95% CI)	OR^b^ (95% CI)^b^
rs16944	GG	GA + GG			
Clinical					
Localized	17	51	0.530	0.714 (0.250, 2.045)	0.686 (0.235, 2.002)
Advanced	7	15			
Gleason					
>7	11	25	0.496	1.388 (0.540, 3.568)	1.404 (0.539, 3.660)
≤7	13	41			
Total PSA (ng/ml)					
>20	12	27	0.442	1.444 (0.565, 3.693)	1.745 (0.654, 4.655)
≤20	12	39			

rs2070874	TT	TC + CC			
Clinical					
Localized	40	28	0.434	0.667 (0.241, 1.847)	0.621 (0.218, 1.770)
Advanced	15	7			
Gleason					
>7	22	14	1.000	1.000 (0.421, 2.375)	1.075 (0.443, 2.607)
≤7	33	21			
Total PSA (ng/ml)					
>20	26	13	0.344	1.517 (0.638, 3.608)	1.505 (0.611, 3.707)
≤20	29	22			

rs2227284	TT	TG + GG			
Clinical					
Localized	52	16	0.938	0.956 (0.305, 3.000)	0.873 (0.270, 2.821)
Advanced	17	5			
Gleason					
>7	28	8	0.839	1.110 (0.407, 3.027)	1.208 (0.431, 3.381)
≤7	41	13			
Total PSA (ng/ml)					
>20	31	8	0.580	1.326 (0.488, 3.605)	1.190 (0.422, 3.360)
≤20	38	13			

rs7175701	TT	TC + CC			
Clinical					
Localized	66	2	1.000	—	—
Advanced	22	0			
Gleason					
>7	36	0	0.515	—	—
≤7	52	2			
Total PSA (ng/ml)					
>20	38	0	0.507	—	—
≤20	50	2			

rs11556218	TT	TG + GG			
Clinical					
Localized	52	16	0.237	1.857 (0.661, 5.221)	1.876 (0.664, 5.302)
Advanced	14	8			
Gleason					
>7	23	13	0.098	0.453 (0.175, 1.169)	0.453 (0.174, 1.176)
≤7	43	11			
Total PSA (ng/ml)					
>20	29	10	0.847	1.097 (0.426, 2.826)	1.118 (0.424, 2.951)
≤20	37	14			

Notes:^a^Two-sided *χ*2 test for the distributions between TT and TT/GG; ^b^adjusting for age and body mass index (BMI); ^c^localized, T1–2N0M0; advanced, T3–4NxMx or TxN1Mx or TxNxM1. Clinical staging according to the international TNM system for prostate cancer.

## Data Availability

The data used to support the findings of this study are available from the author upon request.
